# Prevention Effects of Chain Management on Pressure Ulcers of Hospitalized Patients

**DOI:** 10.1155/2021/6368189

**Published:** 2021-12-11

**Authors:** Jiao Yao, Jie Zhao, Tao Chen, Xuehui Zeng

**Affiliations:** ^1^Zhongshan Hospital Xiamen University, Xiamen 361004, China; ^2^The First Affiliated Hospital of Xiamen University, Xiamen 361001, China

## Abstract

The study focused on the preventive effects of the chain management model on pressure ulcers in the operating room. Sqoop big data collection module is used to collect patient information from various hospital information systems in a distributed manner. The data were from the clinical data center of the Zhongshan Hospital Xiamen University General Hospital, and 268 patients were selected as the research subjects. A chain management model is constructed, concerning the preventive measures, the management of each link, the perioperative pressure ulcer management, and the reporting of pressure ulcers. Then, the two groups were compared for the SAS and SDS scores before and after nursing, the pressure ulcer sites, pressure ulcer reporting rate, pressure ulcer staging, and nursing satisfaction. The results show that it is not that more collection modules will lead to better cluster performance and that the execution delay is caused by MapReduce requiring the JAVA virtual machine, and after reaching a certain point, the increase in the number of tasks will slow down the process, and as data size increases, DataNote has an expanded capability to analyze data. After nursing treatment, the SAS and SDS scores of the two groups of patients were significantly lower than before treatment (*P* < 0.05). The pressure ulcers were mainly distributed in the forehead, mandible, cheeks, front chest, and knees in the two groups, and the difference between the two groups was statistically significant (*P* < 0.05). The total satisfaction of the observation group was 93.28%, and the total satisfaction of the control group was 92.54%. The patients' satisfaction with the chain management model was higher than that of conventional nursing.

## 1. Introduction

Pressure ulcers, also known as pressure injury (PI), are local skin or subcutaneous tissue damage [1]. In 2016, the National Pressure Ulcer Advisory Group (NPUAP) modified this terminology of pressure ulcers to pressure injury, which is a more accurate description of skin injury [2, 3]. PI is the injury of the local skin or soft tissue located at the bone protuberance. It arises from strong and long-term pressure and shear forces, and the tolerance of soft tissue to pressure and shear forces may be affected by the microenvironment, nutrition, perfusion, and comorbidities [4]. NPUAP divides PI into stage-I PI, stage-II PI, stage-III PI, stage-IV PI, nonstage PI, and deep tissue injury. Medical device-related PI and mucosal PI include both open ulcers and deep tissue damage [5]. In recent years, the multidisciplinary combination has increased the complexity of the operation and the hospitalized patients are predominantly affected by pressure ulcers. According to the *Guidelines for the Prevention of Pressure Injury* by NPUAP, the incidence of pressure ulcers is 4.7%–66.0%. The survey results of 12 hospitals in 3 provinces and 9 cities in China showed that the incidence of PI in hospitalized patients reached 0.63% and that the incidence in elderly people over 70 years old reached 1.34% [6]. In Germany, the incidence of PI was 2%–5% from 2010 to 2015, as per a retrospective analysis. Pressure ulcers during surgery not only increase the patient's pain but also prolong the patient's hospital stay and increase medical consumption [7]. Medical staff does not know the cause of pressure ulcers, and patients tend to have pressure ulcers only when they return to the ward after surgery. As a result, they will not be treated until pressure ulcers are formed and it is easy to miss the best time to prevent pressure ulcers. Improper nursing can also lead to infections, seriously threatening the life of the patient [8, 9].

Chain management generates interconnected points according to the law of the development of things and then effectively classifies the information contained in these connection points. It scientifically and reasonably manages the information so that each link can be effective and continuous [10]. Chain management is generally used in the management and operation mechanism of enterprises. At this stage, it has been widely used in many industries. It focuses on the internal logical relationship between each link, and each restricts and depends on each other [11, 12]. Some scholars introduced chain management in skin management and reduced the incidence of PI from 0.023% to 0.019%, below the national average. Cloud computing provides a convenient and on-demand access mode for medical resources. It can quickly schedule, and users can obtain related computing services through minimal interactive work.

Each link in the preventive nursing of pressure ulcers affects the recovery of the patient. Each link has different responsibilities and functions and forms a chain-like relationship based on specific logical relationships and spatial-temporal relationships [13, 14]. The introduction of cloud computing improves resource utilization, reduces system operating costs, and is conducive to constructing green hospitals [15]. Above, in this study, a chain management model is built and applied to the preventive nursing of pressure ulcers. The informatization of medical data effectively promotes the development of the hospital information system and improves the intelligence level of the hospital information system.

## 2. Materials and Methods

### 2.1. Information Management of Medical Data

An overall system architecture is constructed based on the Hadoop medical big data processing system. The overall architecture is shown in Figure 1. The entire flow chart includes 4 major sections of the medical data life cycle, the management plan, the technical plan, and the business system side. The business system side includes the Sqoop ETL module and the Hadoop section, and the overall architecture of the big data processing system uses the Mahout distributed recommendation engine. Ultimately, a closed loop of collection, storage, analysis, and feedback is formed.

### 2.2. Algorithm Design

The Sqoop big data collection module is used to collect patient visit information from various hospital information systems in a distributed manner. According to user preferences, the records are converted into a simple triplet, and *D* represents the total number of triples.

(1) $$\begin{array}{c} <\text{User ID},\text{ Item ID},\text{ Preference}>. \end{array}$$

The similarity between users is calculated based on acquaintance, such as cosine similarity, Euclidean distance, and Pearson's correlation coefficient. Euclidean distance is the true distance between two points in a multidimensional space, calculated as follows.

(2) $$\begin{array}{c} S\left(X,Y\right)=\sqrt{\sum {\left(X_{i}-y_{i}\right)}^{2}}. \end{array}$$

The Euclidean distance similarity is calculated as follows.

(3) $$\begin{array}{c} \text{Sim}\left(X,Y\right)=\frac{1}{1+s\left(x,y\right)}=\frac{1}{1+\sqrt{\sum {\left(X_{i}-y_{i}\right)}^{2}}}. \end{array}$$

The Pearson-related equation is as follows.

(4) $$\begin{array}{c} \rho \left(X,Y\right)=\frac{\mathrm{cov}\left(x,y\right)}{℘x℘y}=\frac{\sum X_{i}y_{i}--\sum X_{i}-y_{i}/D}{\sum X_{i}{}^{2}-\left(\sum X_{i}{}^{2}\right)/D\left(\sum Y_{i}{}^{2}-\left(\sum Y_{i}{}^{2}\right)/D\right)}, \end{array}$$

where *℘x℘y* indicates that the standard deviation and cov(*x*, *y*) are the ratio between the triples.

The cosine value of the included angle is the vector value of two triplets. The equation to measure the difference between the two is as follows.

(5) $$\begin{array}{c} \cos\;\theta =\frac{\sum X_{i}y_{i}}{\sqrt{\sum X_{i}{}^{2}}\sqrt{\sum y_{i}{}^{2}}}. \end{array}$$

Then, the similarity measurement value is calculated.

The measurement methods are expressed as follows.

(6) $$\begin{array}{c} \text{PRECISION}=\frac{\text{TP}}{\text{TP}+\text{FP}},\\ \text{RECALL}=\frac{\text{TP}}{\text{TP}+\text{FN}}. \end{array}$$

Figure 2 is the distributed flow chart of the algorithm. Each step is a complete MapReduce flow chart.

### 2.3. Chain Management Mode of Pressure Ulcers

Figure 3 is the flow chart of the chain management mode of pressure ulcers. First, a team is organized and specifications are formulated. Then, nursing staff are trained for emergency management, ward management, and monitoring management. Operating room management includes during-surgery and postsurgery management. Finally, postoperative follow-up is carried out.

### 2.4. Preventive Measures and Injury Management

Measures to prevent pressure ulcers are mainly based on reducing, alleviating, and redistributing pressure. Appropriate measures can reduce the duration of pressure. Preventive measures also vary from individual to individual, because the operation time and compression site are different between individuals. The main preventive measures include the choice of the support surface, posture care, local skin protection, intraoperative heat preservation, and continuous postoperative follow-up. The support includes general support and local support. The commonly used support surfaces in operating rooms include gel mattresses, alternating pressure mattresses, and foam mattresses. Studies have shown that high-risk patients are recommended to use viscoelastic polymers. When the pressure exceeds the capillary filling pressure, local blood flow may be blocked. The support surface can reduce the interface pressure but cannot reduce the capillary filling pressure. The posture during the operation affects the patient's compression site. Before the surgery, it is necessary to determine the stress point to reduce the occurrence of pressure ulcers. Applying a protective agent to the local skin plays a protective role. Different protective agent materials have different antihypertensive effects. Intraoperative heat preservation includes active heat preservation and passive heat preservation. Active heat preservation is to heat the heating equipment, and the increase in skin temperature is an independent risk factor for pressure ulcers during surgery. Early prevention can reduce the incidence by 50%, and continuous follow-up after surgery is also important.

Figure 4 is the flow chart of the management of PI, including the assessment of the risk of pressure ulcers, seamless management of the transfer, intraoperative management, the nursing management of the ICU patient, and the continuous follow-up.

### 2.5. Perioperative Management

Effective management can reduce the occurrence of perioperative PI. In the conventional model, the nurses do not visit the operating room and there may exist errors when they understand and convey the disease condition, affecting the timely treatment of the disease. Constructing a scientific perioperative chain management model can improve the scientificity and consistency of management and prevent handover errors. Extending operating room nursing to the ward effectively reduces the incidence of pressure ulcers in the operating room.  Figure 5 shows the perioperative PI chain management, including the organization chain and the link chain. The organization chain includes the organization of the team, systematic training, improvement of supervision and incentive mechanism, and construction of information sharing platform. The link chain includes the intraoperative dynamic evaluation and prevention, seamless postoperative transfer and handover, and continuous follow-up. The preoperative, intraoperative, and postoperative evaluations ensure the comprehensiveness of the handover content and the continuity of preventive measures and achieve continuous tracking of patients. The establishment of the organizational chain ensures the integrity of the entire nursing process and the timeliness and accuracy of treatment.

### 2.6. Reporting of Pressure Ulcers

If a patient develops pressure ulcers during the operation, the nurse in the operating room should immediately report it to the leader of the wound nursing team, the surgeon, and the head nurse. Then, the head nurse will report it to the nursing department, ward, and the responsible nurse through the hospital information system. The reporting time to the nursing department should be controlled within 24 hours. Next, as shown in Figure 6, the nurses evaluate the degree of PI taking into account the intraoperative nursing condition, the shift time, the specific reporting time, and the clarity of the report.

### 2.7. Data Sources

The experimental data all come from the Zhongshan Hospital Xiamen University National Natural Science Gene Project, with Zhongshan Hospital Xiamen University as a cooperator. The medical system used by the hospital is Oracle11 g database and the experimental data are true and reliable. This study collected relevant data of patients in Zhongshan Hospital of Xiamen University from January 1, 2000, to January 1, 2015. A total of 189,340 patients were involved, and finally, 268 patients under the inclusion criteria of this study were selected as the research subjects, including 128 men and 140 women, with an average age of (45,82 ± 2.18). Inclusion criteria are as follows: (I) 18–80 years old; (II) operation time> 2 hours; (III) patients voluntarily signed an informed consent form; and (IV) no PI before the surgery. Exclusion criteria are as follows: (I) those with incomplete clinical data; (II) those who did not voluntarily participate in this research; (III) those with heart, liver, and kidney dysfunction; and (IV) patients with mental illness. In this study, patients were divided into two groups according to random numbers. In the control group, there were 134 cases, including 86 women and 48 men, aged 26–78 years old, with an average age of (43,6 ± 2.9) years. In the observation group, there were 134 cases, including 92 women and 42 men, aged 27–76 years old, with an average age of (42,2 ± 3.6) years. The difference between the two groups of patients was not statistically significant (*P* > 0.05). The control group used a conventional management plan, and the observation group used the chain management mode. For the sake of no harm to patients, the data were kept confidential and used only for this research and not for other purposes. The two groups were compared for general information, such as the name, age, height, weight, education level, hypertension, diabetes, preoperative Braden score, operation time, patient's physical activity, intraoperative blood loss, and the occurrence of pressure ulcers within 6 days after the surgery.

Subsequently, the user credibility attributes are summarized based on user ID, user operation time, login range, and operation frequency and operation attributes of the data. Next, the data are standardized as follows.

(7) $$\begin{array}{c} {\hat{X}}_{IJ}=\frac{xin-\bar{x}n}{\sqrt{D\left(xn\right)}}, \end{array}$$

where D(xn) represents the standard deviation of the *n*th attribute, and $\bar{x}n$ represents the mean value of the *n*th attribute in the sample.

The Braden pressure ulcer assessment scale and the Norton scale assist in more accurately predicting the risk of pressure ulcers in clinical work.

The Braden pressure ulcer assessment scale is the most widely used pressure ulcer assessment scale in the world. As shown in Table 1, this scale contains 6 *a* items, namely, nutritional status, activity, mobility, feeling, humidity, friction, and shear force.  Table 2 shows the scores of corresponding degrees of risk for pressure sores.

As shown in Table 3, the Norton scale uses Liker 4 to evaluate the 5 risk factors of pressure ulcers, namely, physical condition, mental condition, activity, mobility, and incontinence. The total score is between 5 and 20. A lower score indicates a greater pressure ulcer risk. Normally, the Norton dose is used for pressure ulcer risk assessment in elderly patients.

### 2.8. Evaluation Index

A questionnaire is designed based on the *Press Ulcer Prevention and Treatment Quick Guide* issued by NPUAP in 2010 and Pressure Ulcer Grading Guidelines issued in 2007, with a total score of 100 points. As shown in Table 4, the questionnaires factor into four aspects: service attitude, nursing operation, health education, and overall impression. The total score of each aspect is 100 points. A score below 80 indicates dissatisfaction, and a score above 80 indicates satisfaction.

The self-depression scale (SDS) and self-rating anxiety scale (SAS) are used to score emotions. A higher score indicates a greater degree of anxiety and depression. There are four grades, namely, very satisfied, generally satisfied, uncertain, and dissatisfied. Overall satisfaction means the sum of very satisfied and generally satisfied.

The perioperative injury staging standard is shown in Table 5. As for nonstaging, it manifests as full-skin and tissue loss, and the degree of injury is concealed. Deep tissue injury and medical device-related PI can be staged according to the standard in Table 5. Mucosal PI cannot be staged.

Next, the incidence of pressure ulcers during the perioperative period is calculated, and the report rate of perioperative pressure ulcers the number of cases reported to the nursing department shall prevail.

### 2.9. Statistical Analysis

All data were processed using SPSS 21.0 statistical software. The measurement data were expressed as ‾*x* ± *s,* and the *t*-test was used. The count data were expressed as a percentage (n, %), and *P* < 0.05 indicated that there was a statistical difference.

## 3. Results

### 3.1. Data Analysis

Faced with a small size of data, the single-node algorithm is even faster than distributed algorithm. This is because there will be time consumption to start MapReduce. As the data size increases, the single-node algorithm cannot complete the processing and analysis of the data within the set time. At this time, the distributed algorithm shows advantages. As shown in Figure 7(a), as data size increases, DataNote has an expanded capability to analyze data.

Figure 7(b) shows the transmission time and total time consumption. The execution delay is caused by MapReduce requiring the JAVA virtual machine. After reaching a certain point, the increase in the number of tasks will slow down the process.

### 3.2. Comparison of General Information

The two groups were compared for the general data. As shown in Table 6, the two groups were mainly distributed between 26 and 78 years old patients. Patients older than 70 years accounted for 17.16% in the observation group and 14.18% in the control group. In terms of education level, elementary students accounted for 56.72% in the observation group and 49.25% in the control group. There are four ways of admission: support by others, wheelchair, flat car, and walking. Walking patients accounted for 76.12% in the observation group and 67.91% in the control group. Limb mobility is divided into mild, moderate, and severe. Mild patients accounted for 83.58% in the observation group and 81.34% in the control group. Smokers accounted for 38.81% in the observation group and 32.09% in the control group. The operation parts include the thoracic spine, cervical spine, and lumbar spine. Patients who had surgery in the lumbar spine accounted for 88.81% in the observation group and 80.60% in the control group. In the observation group, patients whose operation time was less than 4 hours accounted for 88.06%, and patients whose operation time was 4 hours or more accounted for 11.94%. In the control group, patients whose operation time was less than 4 hours accounted for 85.07%, and patients whose operation time was 4 hours or more accounted for 14.93%. The general baseline data of the two groups were not statistically different, and they were comparable (*P* > 0.05).

### 3.3. SAS and SDS Scores

Figure 8 shows the SAS and SDS scores of patients before and after nursing. After nursing treatment, the SAS and SDS scores of the two groups of patients were significantly lower than those before treatment (*P* < 0.05), indicating that the anxiety and depression of the patients after nursing were improved, but the reduction in the observation group was significantly higher than that in the control group.

### 3.4. Stages of Pressure Ulcers

A total of 186 cases had perioperative pressure ulcers in the two groups. There were 76 cases in the control group, of whom 36 cases were in stage I, accounting for 47.37%, 30 cases in stage II, accounting for 39.47%, and 10 cases in stage III, accounting for 13.16. %. There were 110 cases in the observation group, of whom there were 82 cases in stage I, accounting for 74.55%, 21 cases in stage II, accounting for 19.09%, and 7 cases in stage III, accounting for 6.36%. As shown in Figure 9, there were no cases of pressure ulcers of more than stage 4 in the two groups. The difference between the two groups was not statistically significant (*P* > 0.05).

### 3.5. Pressure Ulcer Reporting Rate

The two groups were compared for the reporting rates of perioperative pressure ulcers. As shown in Figure 10, there were a total of 186 cases of perioperative pressure ulcers in the two groups. There were 76 cases in the control group, and 15 cases were not reported and 59 cases were reported. There were 110 cases in the observation group, and 110 cases were reported.

### 3.6. Comparison of Pressure Ulcer Sites

The pressure ulcers in the two groups mainly occurred in the forehead, jaw, cheeks, chest, and knees. It can be seen from Figure 11 that the cases having pressure ulcers in the forehead accounted for the largest portion. In the observation group, those having pressure ulcers in the forehead accounted for 28.36% and those in the control group accounted for 14.18%; those having pressure ulcers in the low jaw accounted for 8.96% in the observation group and those in the control group accounted for 7.46%; those having pressure ulcers in the front chest area accounted for 10.45% in the control group; and those having pressure ulcers in the knee accounted for 5.22% in the observation group and those in the control group accounted for 5.97%. The difference between the two groups was statistically significant (*P* < 0.05).

### 3.7. Nursing Satisfaction

Nursing satisfaction was divided into four aspects: very satisfied, generally satisfied, uncertain, and dissatisfied. As shown in Figure 12, there were 102 very satisfied people in the observation group, accounting for 76.12%, 23 satisfied people, accounting for 17.16%, 6 people holding an uncertain attitude, accounting for 4.48%, and 3 dissatisfied people, accounting for 2.24%. In the control group, 96 people were very satisfied, accounting for 71.64%, 28 were generally satisfied, accounting for 20.90%, 5 were uncertain, accounting for 3.73%, and 5 were dissatisfied, accounting for 3.73%. The overall satisfaction of the observation group was significantly higher than that of the control group, indicating that chain management was more satisfying.

## 4. Discussion

If local tissue of the body is under pressure for a long time, the blood circulation in the body will be obstructed, which leads to skin injury. When tissue lacks nutrients, local tissue will be ruptured and necrotic and such a phenomenon is called pressure ulcers [16, 17]. The existence of pressure ulcers in the operating room not only affects the quality of the operation but also causes depression of the patient's mood, which is not conducive to the recovery of the patient, increases the patient's hospital stay, and increases the medical burden. At the same time, it also increases the economic burden. The patient lacking knowledge about pressure ulcers will be worried about adverse reactions during the operation, which will increase the psychological burden, anxiety, and depression and affect the treatment to a certain effect [18, 19]. In the study, the SAS and SDS scores of patients before and after nursing were analyzed. It was noted that after nursing treatment, the SAS and SDS scores of the two groups of patients were significantly lower than those before treatment (*P* < 0.05), indicating that the anxiety and depression of the patients after nursing were improved, but the reduction in the observation group was significantly higher than that in the control group, which also suggested that patients were anxious and depressed before treatment. Jin et al. (2019) [20] analyzed limb injury and the SAS and SDS scores. Multivariate logistic analysis showed that the anxiety and depression scores before limb injury were high but decreased after surgery. Kulik et al. (2019) [21] studied the prevalence, location, and clinical factors of pressure ulcers. It was found that the prevalence of hospital-acquired pressure ulcers was 9.7%, and about 7.5% was related to medical devices. These data can be used to guide practice and targeted interventions to reduce the risk of PI. In this study, it was found that 186 cases had perioperative pressure ulcers in the two groups. There were 76 cases in the control group, of whom 36 cases were in stage I, accounting for 47.37%, 30 cases in stage II, accounting for 39.47%, and 10 cases in stage III, accounting for 13.16. %. There were 110 cases in the observation group, of whom there were 82 cases in stage I, accounting for 74.55%, 21 cases in stage II, accounting for 19.09%, and 7 cases in stage III, accounting for 6.36%. There were no cases of pressure ulcers of more than stage 4 in the two groups. The difference between the two groups was not statistically significant (*P* > 0.05).

Chain management has been widely used in medical nursing, and some scholars have established a chain management system for PI under the medical consortium mode, which has effectively increased the risk assessment rate of nurses and the implementation rate of preventive measures, and the incidence of pressure sores is significantly decreased. Chain management includes organizational chain and link chain, which can not only realize the vertical management of patients but also ensure the horizontal management, and effectively makes up for the deficiencies in the previous management process. Chain management requires teamwork. Every link, such as the intensive care unit and the ward, is intertwined and inseparable. Only mutual supervision between departments can effectively improve the nursing effect. Wang and Jie (2020) [22] found that chain management has shown good results in the management of the medical field. Supply chain risk management strategies play an important role in supporting the development of enterprises. It provides a reference for drug chain management. The chain management model constructed in this study also shows a positive effect on the prognostic nursing of patients with pressure ulcers. Compared with conventional methods, patient satisfaction is significantly improved, which helps patients recover as soon as possible.

## 5. Conclusions

In this study, the chain management model is applied to the nursing and treatment of pressure ulcers and it effectively reduces the incidence of PI during the perioperative period. The total satisfaction of the observation group was 93.28%, and the total satisfaction of the control group was 92.54%. The patient's satisfaction with the chain management model was higher than that of conventional nursing. It provides a new model for clinical perioperative nursing of pressure ulcers. However, patients in the study are from the same hospital and the results may be affected by mechanical equipment. Additionally, each nurse has inconsistent knowledge of pressure ulcer nursing, which may increase the error during the nursing. In the future, doctors and other team members can be tested for nursing knowledge to achieve better long-term effects.

## Figures and Tables

**Figure 1:** Medical big data information management.

**Figure 2:** Algorithm implementation flow chart.

**Figure 3:** Schematic diagram of chain management of pressure ulcers.

**Figure 4:** Pressure ulcer prevention management and link management.

**Figure 5:** The chain management of pressure ulcers during the perioperative period.

**Figure 6:** Flow chart of the reporting of pressure ulcers.

**Figure 7:** Big data analysis-based performance comparison results.

**Figure 8:** Comparison of SAS and SDS scores (∗ indicated that the difference was statistically significant).

**Figure 9:** Staging of pressure ulcers.

**Figure 10:** Pressure ulcer reporting rate.

**Figure 11:** Comparison of pressure ulcer sites.

**Figure 12:** Comparison of nursing satisfaction.

**Table 1:** Braden pressure ulcer assessment scale.

Project	1 point	2 points	3 points	4 points
Feel damp activity mobility nutrition friction and shear	Completely restricted	Very restricted	Mildly restricted	Undamaged
	Persistent moisture	Very humid	Occasionally wet	Seldom wet
	Bedridden	Confined to chair severely restricted, and it may not be enough to have potential problems	Walk occasionally, mildly restricted, appropriate, and no obvious problems	Walk often
	Cannot at all very bad			Unrestricted
	Has a problem			Good

*Note.* Maximum 23 points and minimum 6 points.

**Table 2:** Questionnaire about pressure ulcer-related knowledge.

	Project	Score
Item rating	Mildly dangerous	15-16
	Moderately dangerous	13-14
	Highly dangerous	10–12
	Extremely dangerous	9 or less

**Table 3:** Norton scale.

Factor	1	2	3	4
Physical condition	Serious	Unstable	Stable and balanced nutrition	Stable and good nutrition
Mental condition	Completely unresponsive	Occasionally unresponsive	Barely unresponsive	Responsive
Activity	Unable to get out of bed	Able to sit	Able to walk under assistance	Able to walk by himself
Mobility	Unable to move	Able to move a little under assistance	Able to move under assistance	Able to move by himself
Incontinence	Incontinence	3–6times/day	1-2times/day	Self-control

*Note.* Maximum 23 points and minimum 6 points.

**Table 4:** Questionnaire about pressure ulcer-related knowledge.

	Project	Score
Related information	Definition of pressure ulcers	10 points
	Staging	20 points
	Risk factors	20 points
	Prevention	20 points
	Treatment measures	40 points
	Health education	100 points
	Nursing operation	100 points
Questionnaire	Overall impression	100 points
	Service attitude	100 points
Satisfaction	≥80	Satisfaction
	＜80	Dissatisfaction

**Table 5:** Staging of perioperative PI.

	Staging	Standard
Stages of pressure injury	I	Skin is intact, erythema that does not whiten by finger
	II	Partial loss of cortex with exposed dermis
	III	Full-thickness skin is missing, and subcutaneous fat tissue, wound edge involute, and granulation tissue can be seen
	IV	Absence of full-thickness skin and tissue, fascia, bones, muscles, ligaments can be seen, and involutions, sinuses, and sneaking are often seen

**Table 6:** Comparison of general information.

Project	Variable	Observation group (%) *N* = 134	Control group (%) *N* = 134	*P*
Gender Age Cultural level	Male	42 (31.34)	48 (35.82)	0.876
	Female	92 (68.66)	86 (64.18)	
	＜70	111 (82.84)	115 (85.82)	
	≥70 University and above high school Junior high school	23 (17.16)	19 (14.18)	0.887
		24 (17.91)	11 (8.21)	
		11 (8.21)	21 (15.67)	
		23 (17.16)	36 (26.87)	
	Primary school	76 (56.72)	66 (49.25)	
Admission method	Support	15 (11.19)	9 (6.72)	
	Wheelchair	8 (5.97)	11 (8.21)	
	Flatcar	9 (6.72)	23 (17.16)	2.908
	Walk	102 (76.12)	91 (67.91)	
Limb mobility	Normal/mild	112 (83.58)	109 (81.34)	
	Moderate	18 (13.43)	22 (16.42)	-0.816
	Severe	4 (2.99)	3 (2.24)	
Smoking	No	52 (38.81)	43 (32.09)	
	Have	82 (61.19)	91 (67.91)	
Surgical site	Thoracic	19 (14.18)	5 (3.73)	
	Cervical spine	11 (8.21)	21 (15.67)	
	Lumbar spine	119 (88.81)	108 (80.60)	
Operation time (H)	<4	118 (88.06)	114 (85.07)	
	≥4	16 (11.94)	20 (14.93)	

## Data Availability

The simulation experiment data used to support the findings of this study are available from the corresponding author upon request.
